# Low Expression of miR-491-3p Is Correlated with Lymph Node Metastasis in Gastric Cancer

This article has been retracted.

**DOI:** 10.1155/2022/7807956

**Published:** 2022-06-30

**Authors:** Haiou Yu, Shuang Luo

**Affiliations:** Department of Gastroenterology, Pingyang Hospital Affiliated to Wenzhou Medical University, Wenzhou, China

## Abstract

**Objective:**

MiR-491-3p, as a tumor suppressor miRNA, was found decreased in many solid tissues. In this study, we aim to investigate miR-491-3p expression in gastric cancer with or without lymph node metastasis (LNM).

**Methods:**

GSE173215 dataset from Gene Expression Omnibus (GEO) was used to measure miRNA expression from tissue samples of gastric cancer patients. Moreover, gastric tumor tissues (non-LNM: *n* = 78; LNM: *n* = 68) were obtained to detect the miR-491-3p expression. Receiver operating characteristic (ROC) curve and Kaplan–Meier (KM) survival analysis, as well as Cox regression analysis, were performed to reveal the role of miR-491-3p in diagnosis and prognosis of gastric cancer.

**Results:**

According to GSE173215 datasets (*t* = −11.25, adjust *P* value = 1.30E-06) and our clinical results (0.390 ± 0.193 vs. 0.562 ± 0.166, *P* < 0.005), the gastric cancer patients with LNM showed lower miR-491-3p expression than those without LNM, demonstrating a high diagnostic efficiency (sensitivity: 74.36%; specificity: 69.12%). In addition, both LNM and low miR-491-3p expression were correlated with the poor prognosis of gastric cancer. Furthermore, the LNM patient with low expression of miR-491-3p had the worse prognosis, but the non-LNM patient with high expression of miR-491-3p had the best prognosis. MiR-491-3p expression (HR = 0.003, 95%CI: 3.35E-04∼0.028) and LNM (HR = 2.326, 95%CI: 1.046∼5.173) were independent risk factors for gastric cancer.

**Conclusion:**

Downregulated miR-491-3p expression was found in gastric cancer, being a high diagnostic efficiency and an independent risk factor for gastric cancer, especially in those having LNM.

## 1. Introduction

As the fifth most common cancer (estimated number of new cases: 1,089,103) and the fourth leading cause of cancer-related death (estimated number of deaths: 768,793) in 2020 (worldwide, both sexes, all ages), gastric cancer is still an important global healthcare problem (https://gco.iarc.fr/today/home). Lymph node metastases (LNM), an intermediate metastatic step from the primary site to the lymph nodes, represent an aggressive yet curable state for many solid tumors [1, 2]. Although LNM was the direct reason for distant metastases, it reflects the biological selection of more aggressive subpopulations showing close relation with local and/or regional recurrence [3, 4]. As demonstrated by many researchers, the presence of LNMs is associated with decreased postoperative survival in gastric cancer [5, 6], being the most important prognostic factors [7]. Because the increased rate of early detection in gastric cancer can lead to an improved prognosis, the concentrations on improving patients' quality of life and utilizing minimally invasive treatments have increased [8].

Recently, in tumor cells, the dysregulation of microRNAs (abbreviated as miRNAs or miRs), as an abundant class of endogenous noncoding RNAs (about 18∼24 nt) suggests their tumorigenic or antitumorigenic effects on target genes expressed in the tumor environment [9, 10]. Several miRNAs were showed to be related to the development and progression of gastric cancer, which also could predict the status of LNM before the surgical operation [11]. For example, Wang *et al.* found the expression of hsa-miR-337-3p and hsa-miR-134 was downregulated in these LMN tissues when compared to primary tumor tissues [12]. Besides, Shin JY *et al.* revealed a downregulation of miR-135a in gastric cancer as an independent risk factor for LNM [8]. Furthermore, miR-1207-5p as one of the ten miRNAs expressed significantly different among gastric cancer patients with or without LNM via miRNA microarray, which could serve as a useful biomarker in the prediction of LNM [13]. MiR-491-3p, a tumor suppressor miRNA, was found decreased in many solid tissues, including brain tumor [14], colorectal cancer [15], and retinoblastoma [16]. It was worth mentioning that miR-491-3p was downregulated in gastric cancer [17]. However, whether the relationship between the dysregulated miR-491-3p and LNM in gastric cancer is still unknown. Therefore, we analyzed the GSE173215 dataset obtained from Gene Expression Omnibus (GEO) by measuring miRNA expression profiles of gastric cancer patients with or without LNM. Furthermore, the miR-491-3p expression was compared between the non-LNM cancer tissues and LNM cancer tissues in clinic to further determine its value of diagnosis and prognosis in gastric cancer.

## 2. Materials and Methods

### 2.1. MicroRNA Microarray in Tumor Tissues

The GSE173215 dataset was obtained from Gene Expression Omnibus (GEO, https://www.ncbi.nlm.nih.gov/geo/query/acc.cgi?acc=GSE173215, platform GPL25134). The expression of miRNA detected using microarray assay with the Agilent-070156 Human_miRNA_V21.0_Microarray 046064 in cancer tissues of gastric cancer patients with or without different lymph node stages was compared based on TNM stage [18]. N0 indicated no LNM (*n* = 10, female/male: 5/5, age range: 39–64 years) and N3 indicated 7 or more LNM (*n* = 10, female/male: 5/5, age range: 45–69 years).

### 2.2. Clinical Samples

After excluding the individuals received preoperative chemotherapy and/or radiation therapy, this study enrolled the 146 subjects with gastric cancer who received curative gastrectomy (male/female: 103/43; average age: 58.3 ± 11.7 years). The samples were consisted of 146 cases of tumor tissues (non-LNM group: *n* = 78; LNM group: *n* = 68 cases), as well as 65 cases of normal gastric mucosa tissues (control group) which were adjacent to cancer in the LNM group. According to the Borrmann type [19], 14 patients were in stage I, 45 in stage II, 51 in stage III, and 32 in stage IV. Furthermore, tumor histological type was assessed according to Lauren's classification [20], and there were 10 cases in high grade, 47 cases in moderate grade, and 89 cases in poor grade among the enrolled participants.

### 2.3. Real Time PCR (qPCR)

Tissue total RNA was reversed using TRIzol Plus RNA purification kit (catalog #: 12183555, Invitrogen, USA), which was then transcribed into cDNA using TaqMan Advanced miRNA cDNA kits (catalog ^#^: A28007, Applied Biosystems), followed by PCR using the TaqMan™ MicroRNA assay (catalog ^#^: 4427975) on an ABI 7500 Realtime PCR system (both from Applied Biosystems). The premiers are listed as follows: miR-491-3p: forward: 5′-CTTATGCAAGATTCCCTTCTA-3′, reverse: 5′-GTG CAGGGTCCGAGGT-3′; U6: forward: 5′- GGACTTTG AAACCCCTTCCTC-3′, reverse: 5′- TTGGACTCGATACACCCCAGG-3′. MiR-491-3p expression levels were normalized and calculated using U6 and 2^−ΔΔCt^, respectively.

### 2.4. Follow-Up Status

The outcome in this study was 5-year overall survival (OS), which was defined as the period from the time of initial diagnosis to the time of death from any cause or survival at the last follow-up.

### 2.5. Statistical Analysis

Data were analyzed using GraphPad Prism Software version 6.0 (GraphPad Software Inc., La Jolla, USA). Student's *t*-test, *χ*^2^ test, or Fisher's exact test were performed to compare differences between two groups as and when appropriate, and ANOVA analysis to compare differences among three groups followed by Tukey's test. The diagnosis and prognosis values of miR-491-3p expression in gastric cancer patients were analyzed using a receiver operating characteristic (ROC) analysis and a Kaplan–Meier (KM) survival analysis with the log-rank (Mantel–Cox) test, respectively. GraphPad prism was also utilized to create univariable and multivariable Cox proportional hazard models using a two-sided *P* < 0.05 as statistical significance.

## 3. Result

MicroRNA microarray revealed the downregulated miR-491-3p in gastric cancer patients with LNM.

According to GSE173215 datasets (Table 1, Figure 1), the gastric cancer patients with 7 or more LNM (LNM group) showed a lower expression of miR-491-3p (*t* = −11.25, adjust *P* value = 1.30E-06), miR-6781-5p (*t* = −5.19, adjust *P* value = 4.96E-02), and miR-3185 (*t* = −5.09, adjust *P* value = 4.96E-02) than those without LNM (non-LNM group), and the most obvious difference of miR-491-3p expression was found between these two groups, which was further explored in our clinical experiment.

MiR-491-3p level descended stepwise from normal to non-LNM cancer to LNM cancer tissues.

As shown in Table 2, a total of 146 patients were evaluated, and most patients were men (*n* = 103, 70.55%). All the patients were further pathologically categorized into the non-LNM group (N0, *n* = 78) and LNM group (N1-3, *n* = 68). The age, gender, Borrmann type, tumor differentiation, and tumor diameter were comparable between the LNM group and non-LNM group (all *P* > 0.05). The result illustrated in Figure 2 revealed that miR-491-3p expression exhibited a stepwise decreasing pattern from normal tissues (0.990 ± 0.394) to non-LNM tumor tissues (0.562 ± 0.166) to LNM cancer tissues (0.390 ± 0.193), with statistically significance among these groups (*F* = 90.70, *P* < 0.001). Both the non-LNM and LNM cancer tissues had the evidently downregulated miR-491-3p expression as compared to the normal tissues (both *P* < 0.001), which is much lower in LNM cancer tissues than the non-LNM tumor tissues (*P* < 0.005).

The diagnosis of miR-491-3p expression for LNM in gastric cancer patients.

Based on ROC analysis using normal tissues as the state variable (Figures 3(a) and 3(b)), miR-491-3p expression has a high diagnostic efficiency for both non-LNM and LNM in gastric cancer, with the area under ROC curve (AUC) as 0.844 (95%CI: 0.775∼0.915; *P* < 0.001; sensitivity: 66.15%; specificity: 97.44%) and 0.927 (95%CI: 0.884 ∼0.971, *P* < 0.001; sensitivity: 83.08%; specificity: 88.24%), respectively. Moreover, the ROC curve of gastric cancer without LNM vs. with LNM were obtained by using miR-491-3p expression, and the result showed the corresponding diagnostic efficiency as follows: AUC: 0.752 (95%CI: 0.672∼0.832; *P* < 0.001) with the sensitivity of 74.36% and specificity of 69.12% (Figure 3(c)).

LNM status and miR-491-3p expression were associates with the prognosis of gastric cancer.

The mortality rates of gastric cancer patients were 28.77% (42/146), and the mortality rates between the non-LNM (14.10%) group and LNM group (45.59%) were highly statistically significant (*P* < 0.001). Moreover, the lower miR-491-3p expression was found in gastric cancer patients who died (0.290 ± 0.153) than those who survived (0.559 ± 0.158) (Figure 4(a)). According to the median expression of miR-491-3p in tumor tissues, a total of 146 patients were divided into high expression group (>0.487, *n* = 73) and low expression group (≤0.487, *n* = 73). Using KM survival analysis, both LNM (*χ*^2^ = 22.43) and low miR-491-3p expression (*χ*^2^ = 30.49) were correlated with the poor prognosis of gastric cancer (both log rank *P* < 0.001, Figures 4(b) and 4(c)). Furthermore, the KM curves showing survival time of patients with or without LNM who express different expression of miR-491-3p were analyzed in combination. And the result revealed the LNM patient with low expression of miR-491-3p had the worse prognosis with mortality rates, but the non-LNM patient with high expression of miR-491-3p had the best prognosis (*χ*^2^ = 42.28, log rank *P* < 0.001, Figure 4(d)).

### 3.1. Univariate and Multivariate Cox Regression Analysis

According to the univariate Cox regression analysis (Table 3), the following clinical features including Borrmann type (HR = 2.352, 95%CI: 1.182 ∼ 4.681), tumor differentiation (HR = 2.163, 95%CI: 1.063 ∼ 4.402), tumor diameter (HR = 2.233, 95%CI: 1.197 ∼ 4.164), miR-491-3p expression (HR = 0.001, 95%CI: 1.49E-04 ∼ 0.006), and LNM (HR = 4.541, 95%CI: 2.277 ∼ 9.060) had critical influences on 5-year OS of patients with gastric cancer (all *P* < 0.05). Subsequently, significant parameters mentioned above in the univariate Cox regression analysis were included in the multivariate Cox regression analysis, and the result revealed that miR-491-3p expression (HR = 0.003, 95%CI: 3.35E-04 ∼ 0.028) and LNM (HR = 2.326, 95%CI: 1.046 ∼ 5.173) were independent risk factors.

## 4. Discussion

Recent data highlighted the important role of miRNAs in human cancers, including gastric cancer, providing a novel method for its diagnosis and treatment [21, 22]. MiR-491-3p as reported to act as an antitumor role in many cancers [23, 24]. Moreover, as demonstrated by several studies, decreased miR-491-3p was exhibited in gastric cancer specimen as compared with the normal tissue [17, 25], being consistent with our clinical results. In a previous study, ginsenoside Rh2, an anticancer nutrient, did lower the activity of colon cancer cells, and under its intervention, the cells presented dysregulation of miR-491-3p and metastasis activities [26]. In addition, miR-491-3p was overexpressed in noncancerous tissues compared with its expression in papillary thyroid cancer (PTC) tissues, which inhibited PTC cell migration and invasion possibly via targeting NEAT1_2 and TGM2 [27]. Furthermore, restored miR-491-3p expression was reported to suppress the invasion of osteosarcoma cells by directly targeting *α*B-crystallin (CRYAB) [24, 28] and the metastasis of hepatocellular carcinoma by blocking epithelial-mesenchymal transition and decreasing matrix metalloproteinase-9 levels [29]. All mentioned above indirectly indicated a certain relationship between miR-491-3p and cancer metastasis.

miRNA microarrays have been widely utilized in the investigation of the molecular complexity of gastric cancer and prognostic classification based on miRNA expression profile [30–32]. The expressions of miRNAs detected using microarray assay (GSE173215 dataset from platform GPL25134) by Yu *et al.* revealed that LNM patients showed lower expressions of miR-491-3p, miR-6781-5p, and miR-3185 than non-LNM patients using GEO2R online software, especially miR-491-3p. It is worth mentioning that miR-491-3p overexpression inhibited GC cell invasion and migration induced by SNHG8 [17] and HMGA2 [25]. In our study, we also found miR-491-3p level is much lower in LNM cancer tissues than that in the non-LNM tumor tissues, implying the negative correlation of miR-491-3p expression with LNM in gastric cancer.

A limited number of biomarker signatures are available and their diagnostic accuracy remains inadequate for diagnosing patients with gastric cancer [33]. Using the detection of miRNAs as the valuable and sensible biomarkers are urgently needed for gastric patients, thus complementing endoscopic diagnosis [34]. A retrospective study demonstrated a predictive value of some miRNAs including miR-221, miR-224, miR-520, and miR-375 for a therapeutic effect of chemotherapy based on platinum derivates in gastric cancer [35]. Emiliya Nikolova et al. revealed that miR-491-3p illustrated a good diagnostic potential in brain metastases compared with normal brain tissues, which could distinguish low-grade from high-grade gliomas and brain metastases from low-grade gliomas [14]. Similarly, in our study, miR-491-3p expression has a good diagnostic efficiency for gastric cancer without LNM (sensitivity: 66.15%; specificity: 97.44%) or with LNM (sensitivity: 83.08%; specificity: 88.24%) using normal tissues as the state variable. Moreover, the ROC curve of gastric cancer without LNM vs. gastric cancer with LNM were obtained by using miR-491-3p expression, and the result showed the highly sensitivity and specificity of 74.36% and 69.12%, suggesting miR-491 could be used as a highly accurate diagnostic biomarker in gastric cancer, especially in those with LNM.

The outcomes of various researches have shown that many miRNAs have a positive value for gastric cancer in prognosis [22, 36]. Recent progress in prognosis and treatment has considerably increased the long-term survival for patients with early gastric cancer [10]. For instance, downregulation of miR-451 was associated with worse prognosis of gastric cancer patients [37]. In addition, miR-125a and miR-146a are tumor suppressors showed to be closely related with LNM, indicating that they should be prognostic elements in gastric cancer [38]. In our experiment, both LNM and low miR-491-3p expression were correlated with the poor prognosis of gastric cancer. Furthermore, the LNM patient with low expression of miR-491-3p had the worse prognosis, but the non-LNM patient with high expression of miR-491-3p had the best prognosis. Most importantly, miR-491-3p expression and LNM were independent risk factors for gastric cancer. Consistently, a decreased miR-491 level is correlated with increased metastasis and lower survival rate in osteosarcoma patients. The results indicated that the prognosis role of miR-491 in gastric cancer, especially in those with LNM. We would like to acknowledge a few limitations to the present study. Firstly, larger enrolled patient are required to validate our result and conclusion. Secondly, we did not get matched blood specimens from the patient to find the diagnostic and prognostic effect of circulating miR-491 in gastric cancer. Last but not the least, the *in vitro* and *in vivo* experiments would be performed to find the potential mechanism of miR-491-3p in gastric cancer as time and funding permit, including the downstream target genes and signal pathway.

In conclusion, gastric cancer patients with LNM showed lower expression of miR-491-3p than those without LNM and normal tissues. MiR-491-3p expression not only had a high diagnostic efficiency for gastric cancer but also were negatively correlated with the poor prognosis. Furthermore, the LNM patient with low expression of miR-491-3p had the worse prognosis, but the non-LNM patient with high expression of miR-491-3p had the best prognosis. According to the univariate and multivariate Cox regression analysis, miR-491-3p expression and LNM were independent risk factors for gastric cancer.

## Figures and Tables

**Figure 1:** Downregulated miR-491-3p was found in gastric cancer patients with lymph node metastasis (LNM) based on GSE173215 datasets. Volcano plot (a) and mean difference plot (b) demonstrated differential expression of miRNA in gastric cancer tissues (LNM group vs. non-LNM group); the red dots indicated miR-491-3p, miR-6781-5p, and miR-3185; (c) the expression of miR-491-3p in gastric cancer tissues with LNM (*n* = 10, female/male: 5/5, age range: 45–69 years) and without LNM (*n* = 10, female/male: 5/5, age range: 39–64 years).

**Figure 2:** miR-491-3p level descended stepwise from normal (*n* = 65) to non-lymph node metastasis (LNM) cancer (*n* = 78) to LNM cancer tissues (*n* = 68). Note: ^*∗∗∗∗*^*P* < 0.001 as compared to control group; ^###^*P* < 0.005 as compared to non-LNM group.

**Figure 3:** The diagnosis of miR-491-3p expression in gastric cancer. (a) The diagnosis of miR-491-3p expression for discriminating gastric cancer without lymph node metastasis (LNM) and normal tissues via receiver operating characteristic (ROC) curve; (b) ROC curve for gastric cancer patients with LNM vs. normal tissues; (c) the ROC curve of gastric cancer without LNM vs. gastric cancer with LNM obtained by using miR-491-3p expression.

**Figure 4:** miR-491-3p expression was associated with better prognosis of gastric cancer. (a) The lower miR-491-3p expression was found in gastric cancer patients who died (*n* = 42) than those who survived (*n* = 104), ^*∗∗∗∗*^*P* < 0.001; (b) Kaplan–Meier survival analysis for high expression of miR-491-3p vs. low expression of miR-491-3p and 5-year overall survival (OS); (c) Kaplan–Meier survival analysis of 5-year OS in gastric patients with or without lymph node metastasis (LNM); (d) Kaplan–Meier curves showing survival time of patients with or without LNM who express different expressions of miR-491-3p analyzed in combination.

**Table 1:** The expressions of miR-491-3p, miR-6781-5p, and miR-3185 in gastric cancer tissues with/without LNM (LNM vs. non-LNM).

	Adjust *P* value	*P* value	*t*	Log_2_FC
hsa-miR-491-3p	1.30E-06	5.04E-10	−11.25	−2.586
hsa-miR-6781-5p	4.96E-02	4.69E-05	−5.19	−2.017
hsa-miR-3185	4.96E-02	5.79E-05	−5.09	−2.730

Note: lymph node metastasis (LNM); fold change (FC).

**Table 2:** Demographic characteristics of the gastric cancer patients with LNM and without LNM.

Variables	N	Non-LNM group (*n* = 78)	LNM group (*n* = 68)	*P* value
Gender				
Male	103	60	43	
Female	43	18	25	0.101
Age (years)				
≤60	77	45	32	
>60	69	33	36	0.245
Borrmann type				
I	18	8	10	
II	45	22	23	
III	51	30	21	
IV	32	18	14	0.647
Differentiation				
High	10	6	4	
Moderate	47	22	25	
Poor	89	30	59	0.132
Tumor diameter				
<3 cm	36	20	16	
3 cm–5 cm	44	26	18	
>5 cm	66	32	34	0.527

Note: lymph node metastasis (LNM).

**Table 3:** Univariate and multivariate Cox regression analysis.

	Univariate analysis						Multivariate analysis					
	B	SE	Wald	*P*	HR	95%CI	B	SE	Wald	*P*	HR	95%CI
*Gender*												
Male vs. Female	−0.391	0.318	1.516	0.218	0.676	0.363∼1.261						

*Age (years)*												
<60 vs. ≥60	−0.363	0.309	1.377	0.241	0.696	0.380∼1.275						

*Borrmann type*												
III/IV vs. I/II	0.855	0.351	5.932	**0.015**	2.352	1.182∼4.681	0.203	0.387	0.275	0.600	1.225	0.574∼2.616

*Differentiation*												
Moderate/high vs. poor	0.772	0.363	4.530	**0.033**	2.163	1.063∼4.402	0.147	0.376	0.153	0.695	1.159	0.554∼2.423

*Tumor diameter (cm)*												
≥5 vs. <5	0.803	0.318	6.382	**0.012**	2.233	1.197∼4.164	0.452	0.324	1.948	0.163	1.571	0.833∼2.965
miR-491-3p expression	−6.944	0.954	52.929	**3.46E-13**	0.001	1.49E-04∼0.006	−5.787	1.129	26.275	**2.96E-07**	0.003	3.35E-04∼0.028
LNM vs. non-LNM	1.513	0.352	18.445	**1.75E-05**	4.541	2.277∼9.060	0.844	0.408	4.288	**0.038**	2.326	1.046∼5.173

Note: lymph node metastasis (LNM); standard error (SE); hazard ratios (HR); 95% confidence intervals (95%CI); bold font indicates the parameter showing statistical difference.

## Data Availability

The data used to support the findings of this study are included within the article.
